# Keratin 80 Promotes Migration and Invasion of Non-Small Cell Lung Cancer Cells by Regulating the TGF-*β*/SMAD Pathway

**DOI:** 10.1155/2022/2630351

**Published:** 2022-09-19

**Authors:** Yueyang Tong, Xueyuan Chen, Zhemin Feng, Changqing Xu, Yaqian Li

**Affiliations:** Department of Respiratory and Critical Care Medicine, The Affiliated Hospital of Hangzhou Normal University, Hangzhou, China

## Abstract

Upregulation of keratin 80 (KRT80) expression levels and carcinogenic function has been found in several types of tumors. However, its contribution and mechanism in NSCLC remain to be outlined. In this study, bioinformatic investigation from the TCGA dataset revealed that KRT80 was confirmed to be elevated in human NSCLC tissues. The results of qRT-PCR and Western blot assays disclosed that KRT80 was uplifted in NSCLC cells. Data from CCK-8 and colony formation assays exhibited that depletion of KRT80 restrained NSCLC cell proliferation. Findings from Transwell and Western blot assays illustrated that downregulation of KRT80 inhibited NSCLC cell migration, invasion, and EMT. Further mechanism exploration implied that KRT80 may be included within the regulation of EMT of NSCLC cells by affecting the TGF-*β*/SMAD pathway. Moreover, depletion of KRT80 attenuated xenograft tumor growth and the expressions of KRT80, Ki-67, and TGFBR1. In conclusion, depletion of KRT80 repressed NSCLC cell proliferation, invasion, and EMT, possibly mediated by the TGF-*β*/SMAD signaling pathway, indicating that KRT80 may be a potentially useful target for NSCLC.

## 1. Introduction

Lung cancer is a malignant tumor that debilitates human health and life, with high morbidity and mortality [1, 2]. About 80% to 90% of all lung cancer patients are non-small cell lung cancer (NSCLC) patients [3]. So far, lung cancer patients are mainly treated with multiple combined therapies based on surgery. With the development of medical science and technology, molecular targeted therapy is becoming more and more the first choice for cancer treatment, providing a new approach for early treatment of NSCLC patients [4]. However, the five-year overall survival rate of the majority of lung cancer patients is approximately only 15%, and more than 90% of patients die rapidly due to continuous metastasis of lung cancer cells, and the prognosis is still not satisfactory [5, 6].

Epithelial-mesenchymal transformation (EMT) serves an important function in the metastasis progress of lung cancer cells, and the occurrence of EMT is related to a variety of cytokines, transcription factors, and signal transduction pathways, among which the EMT mediated by TGF-*β* exerts a pivotal role in metastasis and invasion of NSCLC [7, 8]. Polypeptide growth factors secreted by the TGF‐*β* superfamily participated in a variety of pathophysiological processes, including cellular responses, for example, differentiation, proliferation, and migration [9, 10]. TGF-*β* cell signal transduction is finely regulated at different levels, including the regulation of ligands, receptors, SMADs family proteins, and nuclear transcriptional levels [11–13]. TGF-*β* ligand binds and activates TGFBR2. TGFBR2 recruits and binds TGFBR1 to form a TGFBR2-ligand-TGFBR1 heterotrimer [14]. Activated TGFBR1 phosphorylates the SMADs protein family, which leads to signal transduction into cells, thus regulating the expression of target genes and affecting tumor progression [15].

Keratin is a filamentous cytoskeletal protein of epithelial cells that keeps up structural integrity, including two types: acidic (type I) keratin and alkaline (type II) keratin [16, 17]. Keratin 80 (KRT80), located on chromosome 12q13, encodes 452 amino acids and is a type II Keratin [18]. Keratin is a typical epithelial cell marker, widely expressed in sarcoma, trophoblastic tumors, and other tumors, and plays an imperative part in controlling cell migratory and invasive capacities as well as EMT [19–21]. However, the roles and mechanisms of KRT80 were largely unknown in NSCLC.

In the current work, we found that KRT80 was elevated in lung cancer, and depletion of KRT80 repressed the proliferation and invasion of NSCLC cells. Furthermore, exhaustion of KRT80 significantly inhibited TGF-*β*/SMAD signaling pathway. Importantly, rescue assay revealed that TGF‐*β*1 could reverse the suppression of KRT80 knockdown on NSCLC cell progression. Xenograft tumor experiments showed that depletion of KRT80 attenuated xenograft tumor growth in mice.

## 2. Materials and Methods

### 2.1. Cell Culture and Transfection

NSCLC cell lines (HCC827, H1650, A549, and H1299) and lung epithelial cells (BEAS-2B) were obtained from iCell Bioscience Inc (Shanghai, China) and cultured according to the instructions. shRNAs targeting KRT80 (sh-KRT80#1/#2) and sh-NC were cloned into pLKO.1 vector and provided by RiboBio (Guangzhou, China). Cells were transfected for 48 h by Lipofectamine 3000 (Invitrogen, USA).

### 2.2. qRT-PCR Analysis

TRIzol reagent (15596026, Invitrogen, USA) and PrimeScript RT kit (RR014B, Takara, Japan) were used to extract total RNA and reverse transcribe it into cDNA, respectively. SYBR Premix Ex TaqII reagent (RR820A, Takara, Japan) was selected for qRT-PCR analysis on the ABI 7500HT Fast Real-Time PCR System (Applied Biosystems, USA). The primers are listed as follows: KRT80, F: 5′- CCTCCCTAATTGGCAAGGTG -3′; R: 5′- AGATGCCCGAGGTCG AAGAT-3′; GAPDH, F: 5′- GGAGCGAGATCCCTCCAAAAT-3′; R: 5′- GGCTGT TGTCATACTTCTCATGG-3′. The data were normalized to GAPDH and then analyzed based on the 2^−ΔΔCT^ method.

### 2.3. Cell Proliferation Assays

To measure cell viability, 3 × 10^3^ A549 cells were inoculated into 96-well plates. After 24, 48, 72, and 96 hours of incubation, each well was treated with the addition of 10 *µ*L CCK-8 (C0038, Beyotime, China). Cell viability was calculated by detecting absorbance at 450 nm by a microplate reader.

To detect the formation of cell clones, 5 × 10^3^ A549 cells were seeded in 6-well plates and refined for 14 days. Cell clones were fixed and subsequently dyed with crystal violet (C0775, Sigma-Aldrich, USA).

### 2.4. Western Blot

Total proteins were isolated, quantified, and separated by RIPA (P0013 E, Beyotime, China), BCA kit (PC0020, Solarbio, China), and SDS-PAGE, respectively. Following transfer to PVDF membranes, the proteins were obstructed with 5% non-fat milk, and the next step is to incubate with the primary antibodies: KRT80 (ab222325, Abcam, USA), E-cadherin (AF0131, Affinity Biosciences, China), N-cadherin (AF4039, Affinity Biosciences, China), Vimentin (BF8006, Affinity Biosciences, China), TGFBR1 (AF5347, Affinity Biosciences, China), SMAD2 (AF6449, Affinity Biosciences, China), p-SMAD2 (AF3450, Affinity Biosciences, China), SMAD3 (AF6362, Affinity Biosciences, China), p-SMAD3 (AF3362, Affinity Biosciences, China), and GAPDH (AF7021, Affinity Biosciences, China) for 12 h. Immediately afterward, the membranes were subject to incubation with the secondary antibody (A-B6721, Abcam, UK) conjugated with HRP for 2 hours, and the signals were observed with an ECL detection kit (P0018S, Beyotime, China) and quantitated by fragments' intensities using the Image *J* software.

### 2.5. Transwell Assay

24 hours after transfection, 1 × 10^5^ A549 cells were added to 200 *μ*L DMEM medium without serum and cultured in the top chambers. The top chamber prepared with polycarbonate membrane (8 *μ*m pore size, Corning, USA) uncoated or precoated with matrix Matrigel was employed to simulate cell migration or invasion conditions, respectively. In the bottom chamber, 600 *μ*L complete DMEM (containing 10% FBS) was added and thereafter cultivated for 24 hours. Then, after fixing the cells that moved through matrix membrane to the bottom chambers, they were dyed with 0.5% crystal violet, counted numbers, and took pictures.

### 2.6. In Vivo Tumorigenesis Model

Twelve 5-6-week-old BALB/cnude mice were distributed randomly into the sh-NC and sh-KRT80 groups (*n* = 6 per group). 100 *μ*L of cell suspension containing 5 × 10^6^ A549 cells, which were stabilized transfected with sh-NC or sh-KRT80, was administered by subcutaneous injection to each mouse. Tumor sizes were examined at each 3-day interval and measured as volume (mm^3^) = 0.5 × length × width^2^. At 31 days postinjection, tumors were excised from the executed mice and weighed.

### 2.7. Immunohistochemical Analysis

The tissues were fixed, dehydrated by ethanol gradient, embedded, and cut into 4 *μ*M sections. Immunostaining was performed according to the standard protocols by Servicebio with primary antibodies of Ki-67 (AF0198, Affinity Biologicals, China) KRT80 (PA5-98537, Invitrogen, USA) and TGFBR1 (AF5347, Affinity Biologicals, China) at 4°C for 12 h. The sections were next subjected to incubation with the corresponding secondary antibody (ab97080, Abcam, UK) for 30 min at 37°C, followed by staining with DAB (G1212, Servicebio, China) and counterstaining with hematoxylin (G1004, Servicebio, China).

### 2.8. Statistics

There were at least three replications of all experiments conducted independently, and data were processed and analyzed with SPSS 16.0 (SPSS, Chicago, IL). Tukey was utilized to characterize the differences between two groups. One-way ANOVA was used for measurement data among multiple groups. All data were presented as mean ± SD. *P* < 0.05 was defined as a significant difference.

## 3. Results

### 3.1. KRT80 Expression Was Elevated in NSCLC

KRT80 expression in NSCLC tissues was initially investigated by bioinformatics analysis. Analysis of data from the online site UALCAN revealed that KRT80 was dramatically more abundant in primary tumor tissues of lung cell squamous and adenocarcinoma than in normal samples (Figure 1(a)). In addition, the KRT80 level is elevated across cancer stages I–IV and nodal metastasis status N0–N3 in both LUAD and LUSC by the UALCAN algorithm (Figures 1(b)–1(c)). As demonstrated in Figures 1(d)and 1(e), KRT80 mRNA and protein were augmented in NSCLC cells (HCC827, H1650, A549, and H1299) in comparison to BEAS-2B cells. Moreover, the results illustrated that KRT80 was notably more expressed in A549 cells versus other NSCLC cells; thus, A549 cells were selected to transfect siRNA. These results implicated that KRT80 was expressed at an elevated level in NSCLC.

### 3.2. Repressing KRT80 Abrogated NSCLC Cell Proliferation In Vitro

Next, we conducted loss-of-function studies to explore whether KRT80 could regulate the malignant behaviors in NSCLC cells. To this end, two different shRNAs (sh-KRT80#1 and sh-KRT80#2) against KRT80 were constructed and stably transfected into A549 cells. Afterward, qRT-PCR and Western blot were adopted to evaluate the knockdown effect, and apparently, sh-KRT80 #1 had a more promising knockdown outcome and was therefore selected for the following study (Figures 2(a)–2(b)). Subsequently, CCK-8 assays uncovered that depletion of KRT80 visibly arrested the proliferation rate of A549 cells (Figure 2(c)). Consistently, downregulation of KRT80 remarkably reduced colony numbers of A549 cells with respect to the sh-NC group (Figure 2(d)). Collectively, the above findings implied that the depression of KRT80 restrains NSCLC cell proliferation in vitro.

### 3.3. Depletion of KRT80 Impeded NSCLC Cell Migratory and Invasive Abilities as well as EMT

Metastasis is a leading cause of NSCLC lethality. Next, we explored the function of KRT80 in the metastatic characteristics of NSCLC cells. The Transwell assay exhibited that depletion of KRT80 depressed the amount of migrating and invading A549 cells (Figures 3(a)–3(b)). Changes in EMT-relevant proteins were determined (Figure 3(c)), and the results presented that the N-cadherin and Vimentin levels were noticeably declined, and the E-cadherin levels were appreciably enhanced in A549 cells with knockdown of KRT80 than those in the sh-NC group. Together, these findings revealed that depletion of KRT80 impeded NSCLC cell migratory and invasive abilities as well as EMT.

### 3.4. Knockdown of KRT80 Inhibits TGF-*β*/SMAD Signaling in NSCLC Cells

Numerous pieces of evidence confirmed that the TGF-*β*/SMAD as one of the EMT-induced signals in tumor-associated stroma can induce or functionally activate tumor cells [22, 23]. TGF-*β* serves an important role in stimulating epithelial cells to initiate EMT through activating SMAD signaling [24, 25]. Therefore, we focused on the effects of KRT80 on the TGF-*β*/SMAD signaling. Analysis from the online site UALCAN (Figure 4(a)) displayed that KRT80 was a positive correlation with TGFBR1 in adrenocortical carcinoma (ACC), kidney renal papillary cell carcinoma (KIRP), and thyroid carcinoma (THCA), and their Pearson Correlation Coefficient was 0.37, 0.34, and 0.3 [26]. So, we used the Western blot to analyze the protein expression level when the KRT80 was silenced to explore the correlation between it and TGFBR1 in NSCLC cells. Additionally, the data from the Western blot assay illustrated that depletion of KRT80 dramatically diminished the protein levels of TGF-*β*1 and p-SMAD2/3 in A549 cells, whereas SMAD2/3 level was not altered (Figure 4(b)). These data suggested that downregulation of KRT80 suppresses the TGF-*β*/SMAD pathway in NSCLC cells.

### 3.5. KRT80 Regulates the EMT Process of NSCLC Cells by Mediating the TGF-*β*/SMAD Pathway

To determine whether KRT80-induced EMT is mediated through the TGF-*β* pathway, we induced the EMT process in A549 cells with TGF-*β*1, a SMAD2/3 cascade agonist at a concentration of 10 *n*g/ml. The results in Figures 5(a) and 5(b) illustrated that, in A549 cells, depletion of KRT80 notably repressed cell migration and invasion, while TGF-*β*1 treatment had the opposite results. Analysis of changes in EMT-related proteins in A549 cells disclosed that TGF-*β*1 stimulation partially inverted the effects of sh-KRT80 on E-cadherin, N-cadherin, and Vimentin levels (Figure 5(c)). These results manifested that KRT80 regulates EMT in NSCLC cells by triggering activation of the TGF-*β*/SMAD pathway.

### 3.6. Depletion of KRT80 Impeded NSCLC Cell Migratory and Invasive Abilities as well as EMT

For illustrating the contribution of KRT80 in the evolution of NSCLC tumors, we constructed a mouse Xenograft tumor model. As exhibited in Figures 6(a)–6(c), the growth and weight of tumors were discriminately restricted in the KRT80 knockdown mice in contrast to the sh-NC group. Immunohistochemical staining assay (Figure 6(d)) evidenced that Ki-67, KRT80, and TGFBR1 levels were visibly diminished in the sh-KRT80 group in contrast to the sh-NC group. Thus, the above findings implied that depletion of KRT80 inhibits NSCLC xenograft tumor growth in vivo.

## 4. Discussion

Amassing evidence recommends that KRT80 is abnormally communicated in tumor tissues and is correlated with tumor progression. Lin et al. proved that KRT80 level was elevated in colorectal cancer tissues and remarkably correlated with lymph node enlargement and distant metastasis as well as severe pathological staging and confirmed that KRT80 may accelerate tumor growth through the mediation of cell cycle and DNA replication pathway [27]. KRT80 has been implicated in the evolution of breast and gastric cancers [28, 29]. In the current work, we observed that KRT80 was expressed with upregulation in NSCLC tissues and cells and that depletion of KRT80 attenuated the proliferative and invasive potential as well as EMT of NSCLC cells and impeded xenograft tumorigenesis of NSCLC.

KRT80 was previously documented to facilitate the colorectal cancer cell proliferation and invasion through the AKT pathway and interacted with PRKDC [30]. A recent study found that KRT80 accelerates ovarian cancer cell growth, cycle transitions from G1 to S phase, migration, and invasion through activating MEK/ERK pathway [31]. Although the mechanism of KRT80 regulating tumor progression has been gradually reported, the mechanism of KRT80 in NSCLC is still unclear and worth exploring. Keratin 7, a molecule of the keratin family, has been characterized to drive EMT of ovarian cancer cells through the TGF-*β*/SMAD2/3 pathway. Moreover, we found a significant correlation between KRT80 and TGFBR1 in NSCLC by UALCAN data analysis platform. TGFBR1 gene is known to provide instructions for the production of TGF-*β*R I protein [32]. TGF-*β*R I and TGF-*β*R II receptors bind to TGF-*β*, causing phosphorylation and enactment of SMAD2 and SMAD3, forming a trimer with SMAD4 and transporting them to the nucleus, and interacting with other transcription factors [25, 33]. Based on the above findings, we concentrated on the link between KRT80 and TGFBR1-related TGF-*β*/SMAD axis. The findings implied that the knockdown of KRT80 restrained the TGF-*β*/SMAD pathway.

After SMAD trimer translocation, E-cadherin diminished, and N-cadherin and Vimentin were enhanced, thus facilitating EMT in cancer. [11]. In addition, we explored the role of KRT80 on TGF-*β*-mediated EMT. We discovered that the suppressive impacts of sh-KRT80 on NSCLC cell migration, invasion, and EMT were abolished by exogenous TGF-*β*1 stimulation. Accordingly, we demonstrated that KRT80 possibly moderates the progression and evolution of NSCLC by mediating the TGF-*β*/SMAD signaling. Scientists have found that natural products can inhibit the TGF-*β*/SMAD signaling to antagonize the growth and invasion of NSCLC cells. For example, Zhang's team investigated the inhibitory effects of Nagilactone E (NLE) that was isolated from the seeds of *Podocarpus nagi* on NSCLC. They found that NLE inhibited migration and invasion of NSCLC A549 cells by antagonizing the TGF-*β*/SMAD signaling [34]. And Da discovered that Nobiletin from *Citrus depressa* prevented EMT of NSCLC A549 cells by inactivating TGF-*β*/SMAD3 signaling [35]. It suggests that is worthwhile to develop natural products that inhibit KRT80.

To conclude, this work highlighted that downregulation of KRT80 impedes proliferative, invasive capabilities, and EMT of NSCLC cells, possibly via adjusting the TGF-*β*/SMAD pathway. These discoveries extend our understanding of the mechanism of KRT80 and may be an underlying beneficial target for NSCLC, providing basic data for the exploration of the treatment of NSCLC.

## Figures and Tables

**Figure 1:** KRT80 expression was elevated in NSCLC. (a) The expression of KRT80 in primary tumor and normal tissues from the TCGA database were analyzed by UALCAN (http://ualcan.path.uab.edu/analysis.html). (b) UALCAN was utilized to explore KRT80 expression in different stages of NSCLC and normal patients from the TCGA database. (c) UALCAN was utilized to identify the expression of KRT80 from the TCGA database in different grades of NSCLC and normal patients. (d) qRT-PCR recognized KRT80 mRNA. (e) The Western blot estimated KRT80 protein level.  ^*∗*^ ^*∗*^*P* < 0.01 and  ^*∗*^ ^*∗*^ ^*∗*^*P* < 0.001.

**Figure 2:** Repressing KRT80 abrogated NSCLC cell proliferation in vitro. (a and b) KRT80 mRNA and protein in transfected cells were examined using qRT-PCR and Western blot. (c) The viability of A549 cells was estimated by CCK-8. (d) Clones of A549 cells were assessed by colony formation assay.  ^*∗*^ ^*∗*^*P* < 0.01 and  ^*∗*^ ^*∗*^ ^*∗*^*P* < 0.001.

**Figure 3:** Depletion of KRT80 impeded NSCLC cell migratory and invasive abilities as well as EMT. (a and b) The Transwell assay was conducted to measure the number of migrating and invaded A549 cells (Scale bar = 40 *μ*m). (c) The Western blot assessed protein levels.  ^*∗*^ ^*∗*^*P* < 0.01 and  ^*∗*^ ^*∗*^ ^*∗*^*P* < 0.001. Knockdown of KRT80 inhibits TGF-*β*/SMAD signaling in NSCLC cells.

**Figure 4:** Knockdown of KRT80 inhibits TGF-*β*/SMAD signaling in NSCLC cells. (a) The relationship between the expression of KRT80 and TGFBR1 in adrenocortical carcinoma (ACC), kidney renal papillary cell carcinoma (KIRP), and thyroid carcinoma (THCA) was explored using the UALCAN data analysis platform (http://ualcan.path.uab.edu/index.html). (b) The Western blot assessed protein levels in NSCLC cells.  ^*∗*^ ^*∗*^*P* < 0.01 and  ^*∗*^ ^*∗*^ ^*∗*^*P* < 0.001.

**Figure 5:** KRT80 regulates the EMT process of NSCLC cells by mediating the TGF-*β*/SMAD pathway. (a and b) The Transwell assay was conducted to measure the number of migrating and invaded A549 cells (Scale bar = 40 *μ*m). (c) The Western blot assessed protein levels.  ^*∗*^ ^*∗*^*P* < 0.01 and  ^*∗*^ ^*∗*^ ^*∗*^*P* < 0.001. Depletion of KRT80 hinders xenograft tumorigenesis of NSCLC.

**Figure 6:** Depletion of KRT80 hinders xenograft tumorigenesis of NSCLC. (a) The representative representation of tumor nodules. (b) Tumor volume alteration curves in mice. (c) Statistical data of tumor weights of mice. (d) Levels of KRT80, Ki-67, and TGFBR1 in tissue sections of mice tumors were detected using an immunohistochemistry assay (top, bottom panel; scale bar = 100, 50 *μ*m).  ^*∗*^ ^*∗*^*P* < 0.01 and  ^*∗*^ ^*∗*^ ^*∗*^*P* < 0.001.

## Data Availability

The dataset used and analyzed in this study can be obtained from the corresponding author upon reasonable request.

## Additional Points

*Highlights*. (1) The expression of keratin 80 (KRT80) was elevated in NSCLC. (2) Suppression of KRT80 restrained NSCLC cell migratory and invasive abilities as well as EMT. (3) KRT80 facilitated the EMT process of NSCLC cells via activating the TGF-*β*/SMAD pathway. (4) Depletion of KRT80 inhibits NSCLC tumor growth in vivo.

## References

[1] Cheng T. Y., Cramb S. M., Baade P. D., Youlden D. R., Nwogu C., Reid M. E. (2016). The international epidemiology of lung cancer: latest trends, disparities, and tumor characteristics. *Journal of Thoracic Oncology*.

[2] Wang L., Yu C., Liu Y. (2016). Lung cancer mortality trends in China from 1988 to 2013: new challenges and opportunities for the government. *International Journal of Environmental Research and Public Health*.

[3] Zappa C., Mousa S. A. (2016). Non-small cell lung cancer: current treatment and future advances. *Translational Lung Cancer Research*.

[4] Pikor L. A., Ramnarine V. R., Lam S., Lam W. L. (2013). Genetic alterations defining NSCLC subtypes and their therapeutic implications. *Lung Cancer*.

[5] Allemani C., Weir H. K., Carreira H. (2015). Global surveillance of cancer survival 1995–2009: analysis of individual data for 25,676,887 patients from 279 population-based registries in 67 countries (CONCORD-2). *The Lancet*.

[6] Wang X., Adjei A. A. (2015). Lung cancer and metastasis: new opportunities and challenges. *Cancer and Metastasis Reviews*.

[7] Kim B. N., Ahn D. H., Kang N. (2020). TGF-*β* induced EMT and stemness characteristics are associated with epigenetic regulation in lung cancer. *Scientific Reports*.

[8] Thompson J. C., Hwang W.-T., Davis C. (2020). Gene signatures of tumor inflammation and epithelial-to-mesenchymal transition (EMT) predict responses to immune checkpoint blockade in lung cancer with high accuracy. *Lung Cancer*.

[9] Syed V. (2016). TGF-Β signaling in cancer. *Journal of Cellular Biochemistry*.

[10] Jiang X. U. E., Zhang H. (2022). Knockdown of lncRNA XIST prevents the epithelial-mesenchymal transition of TGF-*β*2-induced human lens epithelial cells via miR-124/slug axis. *Biocell*.

[11] Colak S., Ten Dijke P. (2017). Targeting TGF-*β* signaling in cancer. *Trends in Cancer*.

[12] Batlle E., Massagué J. (2019). Transforming growth factor-*β* signaling in immunity and cancer. *Immunity*.

[13] Yu B., Jin X. Q., Yu W. Y., Dong Y. Y., Ying H. Z., Yu C. H. (2021). 1*β*-Hydroxyalantolactone from inulae flos alleviated the progression of pulmonary fibrosis via inhibiting JNK/FOXO1/NF-*κ*B pathway. *International Immunopharmacology*.

[14] Lin E., Kuo P.-H., Liu Y.-L., Yang A. C., Tsai S.-J. (2017). Transforming growth factor-*β* signaling pathway-associated genes SMAD2 and TGFBR2 are implicated in metabolic syndrome in a Taiwanese population. *Scientific Reports*.

[15] Wang J., Xiang H., Lu Y., Wu T. (2021). Role and clinical significance of TGF‑*β*1 and TGF‑*β*R1 in malignant tumors (review). *International Journal of Molecular Medicine*.

[16] Uenishi T., Kubo S., Yamamoto T. (2003). Cytokeratin 19 expression in hepatocellular carcinoma predicts early postoperative recurrence. *Cancer Science*.

[17] Strnad P., Paschke S., Jang K.-H., Ku N.-O. (2012). Keratins. *Current Opinion in Gastroenterology*.

[18] Rogers M. A., Edler L., Winter H., Langbein L., Beckmann I., Schweizer J. (2005). Characterization of new members of the human type II keratin gene family and a general evaluation of the keratin gene domain on chromosome 12q13.13. *Journal of Investigative Dermatology*.

[19] Wu P. C., Fang J. W., Lau V. K., Lai C. L., Lo C. K., Lau J. Y. (1996). Classification of hepatocellular carcinoma according to hepatocellular and biliary differentiation markers. clinical and biological implications. *American Journal Of Pathology*.

[20] Govaere O., Komuta M., Berkers J. (2014). Keratin 19: a key role player in the invasion of human hepatocellular carcinomas. *Gut*.

[21] Omary M. B., Ku N.-O., Strnad P., Hanada S. (2009). Toward unraveling the complexity of simple epithelial keratins in human disease. *Journal of Clinical Investigation*.

[22] O’Connor J. W., Gomez E. W. (2014). Biomechanics of TGF*β*-induced epithelial-mesenchymal transition: implications for fibrosis and cancer. *Clinical and Translational Medicine*.

[23] Lamouille S., Xu J., Derynck R. (2014). Molecular mechanisms of epithelial-mesenchymal transition. *Nature Reviews Molecular Cell Biology*.

[24] Ji Q., Liu X., Han Z. (2015). Resveratrol suppresses epithelial-to-mesenchymal transition in colorectal cancer through TGF-*β*1/smads signaling pathway mediated Snail/E-cadherin expression. *BMC Cancer*.

[25] An Q., Liu T., Wang M. Y. (2021). KRT7 promotes epithelial-mesenchymal transition in ovarian cancer via the TGF-*β*/Smad2/3 signaling pathway. *Oncology Reports*.

[26] Chandrashekar D. S., Karthikeyan S. K., Korla P. K. (2022). UALCAN: an update to the integrated cancer data analysis platform. *Neoplasia*.

[27] Lin J., Fan X., Chen J., Xie X., Yu H. (2020). Small interfering RNA-mediated knockdown of KRT80 suppresses colorectal cancer proliferation. *Experimental and Therapeutic Medicine*.

[28] Song H., Xu Y., Xu T. (2020). CircPIP5K1A activates KRT80 and PI3K/AKT pathway to promote gastric cancer development through sponging miR-671-5p. *Biomedicine & Pharmacotherapy*.

[29] Perone Y., Farrugia A. J., Rodríguez-Meira A. (2019). SREBP1 drives keratin-80-dependent cytoskeletal changes and invasive behavior in endocrine-resistant ER*α* breast cancer. *Nature Communications*.

[30] Li C., Liu X., Liu Y. (2018). Keratin 80 promotes migration and invasion of colorectal carcinoma by interacting with PRKDC via activating the AKT pathway. *Cell Death & Disease*.

[31] Liu O., Wang C., Wang S. (2021). Keratin 80 regulated by miR-206/ETS1 promotes tumor progression via the MEK/ERK pathway in ovarian cancer. *Journal of Cancer*.

[32] Moore-Smith L., Pasche B. (2011). TGFBR1 signaling and breast cancer. *Journal of Mammary Gland Biology and Neoplasia*.

[33] Yang Y. (2021). The role of TGF-beta signaling pathways in cancer and its potential as a therapeutic target. *Evidence-Based Complementary and Alternative Medicine*.

[34] Zhang L. L., Jiang X.-M., Huang M.-Y. (2019). Nagilactone E suppresses TGF-*β*1-induced epithelial-mesenchymal transition, migration and invasion in non-small cell lung cancer cells. *Phytomedicine*.

[35] Da C., Liu Y., Zhan Y., Liu K., Wang R. (2016). Nobiletin inhibits epithelial-mesenchymal transition of human non-small cell lung cancer cells by antagonizing the TGF-*β*1/Smad3 signaling pathway. *Oncology Reports*.

